# Impact of Personal Protective Equipment on Cardiopulmonary Resuscitation and Rescuer Safety

**DOI:** 10.1155/2023/9697442

**Published:** 2023-11-30

**Authors:** Cheng-Hsin Cheng, Ya-Yun Cheng, Mei-Kang Yuan, Yow-Jer Juang, Xuan-Yu Zeng, Chung-Yu Chen, Ning-Ping Foo

**Affiliations:** ^1^Graduate Institute of Medical Sciences, Chang Jung Christian University, Tainan, Taiwan; ^2^Department of Neurosurgery, An Nan Hospital, China Medical University, Tainan, Taiwan; ^3^School of Medicine, College of Medicine, National Sun Yat-sen University, Kaohsiung, Taiwan; ^4^Department of Radiology, An Nan Hospital, China Medical University, Tainan, Taiwan; ^5^Department of Medical Imaging and Radiology, Shu-Zen Junior College of Medicine and Management, Kaohsiung, Taiwan; ^6^Department of Occupational Safety and Health, School of Safety and Health Sciences, Chang Jung Christian University, Tainan, Taiwan; ^7^Occupation Environment and Food Safety Research Center, Chan Jung Christian University, Tainan, Taiwan; ^8^Department of Emergency Medicine, An Nan Hospital, China Medical University, Tainan, Taiwan

## Abstract

**Background:**

High-quality cardiopulmonary resuscitation (CPR) is a key element in the rescue of cardiac arrest patients but is difficult to achieve in circumstances involving aerosol transmission, such as the COVID-19 pandemic.

**Methods:**

This prospective randomized crossover trial included 30 experienced health care providers to evaluate the impact of personal protective equipment (PPE) on CPR quality and rescuer safety. Participants were asked to perform continuous CPR for 5 minutes on a manikin with three types of PPE: level D-PPE, level C-PPE, and PAPR. The primary outcome was effective chest compression per minute. Secondary outcomes were the fit factor by PortaCount, vital signs and fatigue scores before and after CPR, and perceptions related to wearing PPE. Repeated-measures ANOVA was used, and a two-tailed test value of 0.05 was considered statistically significant.

**Results:**

The rates of effective chest compressions for 5 minutes with level D-PPE, level C-PPE, and PAPRs were 82.0 ± 0.2%, 78.4 ± 0.2%, and 78.0 ± 0.2%, respectively (*p* = 0.584). The fit-factor test values of level C-PPE and PAPRs were 182.9 ± 39.9 vs. 198.9 ± 9.2 (*p* < 0.001). The differences in vital signs before and after CPR were not significantly different among the groups. In addition, the fatigue and total perception scores of wearing PPE were significantly higher for level C-PPE than PAPRs: 3.8 ± 1.6 vs. 3.0 ± 1.6 (*p* < 0.001) and 27.9 ± 5.4 vs. 26.0 ± 5.3 (*p* < 0.001), respectively.

**Conclusion:**

PAPRs are recommended when performing CPR in situations where aerosol transmission is suspected. When PAPRs are in short supply, individual fit-tested N95 masks are an alternative. This trial is registered with NCT04802109.

## 1. Introduction

High-quality cardiopulmonary resuscitation (CPR) is a key element in rescuing patients from sudden cardiac death. According to the 2015 American Heart Association guidelines, high-quality CPR includes chest compression that requires a depth between 5 and 6 cm, a rate between 100 and 120 compressions per minute, complete chest recoil, and correct hand position [1]. However, while performing CPR in complex situations, such as exposure to biohazardous aerosol transmission [2–4], chemical agents [5], or during transportation [6], these recommendations are difficult to achieve.

In the past, the Ebola virus epidemic in West Africa caused many infections and deaths in medical personnel. In these circumstances, experts have especially emphasized the importance of personal protective equipment (PPE) [2]. There were also rescuers in Korea being infected by Middle East respiratory syndrome coronavirus while performing CPR [3]. At present, the world is facing enormous challenges. The new coronavirus disease (COVID-19), identified at the end of 2019, caused a worldwide pandemic. As of 4 October 2023, more than 771 million individuals were reported to have been infected with COVID-19, of whom over 6.96 million died, with an overall mortality rate of 0.90% [7]. Among these individuals, many were health caregivers who were exposed to COVID-19 through their work, especially through exposure to aerosol generation procedures (AGPs), and were at a higher risk of infection. WHO has categorized CPR as an AGP that requires the wearing of respirator masks such as N95 masks, powered air-purified respirators (PAPRs), and other types of PPE [8, 9]. While wearing an N95 mask, the fit factor (FF) should be checked before use. The FF is the quantitative ratio of substance concentration in the ambient air versus inside the respirator that is being worn. According to the Occupational Safety and Health Administration (OSHA), adequate protection with the N95 mask is defined as an FF score of ≥100 [10].

However, regarding the impact of PPE on CPR quality, the advantages and disadvantages of different types of PPE on rescuer safety remain unclear and the number of studies in this area is limited [11–17]. Hence, this study was performed to evaluate the impact of different types and levels of PPE on CPR quality and rescuer safety.

## 2. Materials and Methods

### 2.1. Study Design

This simulation study was designed as a prospective randomized crossover trial performed from 1 April 2021 to 30 June 2021 at Annan Hospital, China Medical University, Tainan, Taiwan. The participants were required to perform five minutes of continuous CPR on a Laerdal manikin QCPR (Laerdal, Norway) in the kneeling position while using three types of PPE separated by 120 minutes. The AHA recommends changing rescuers every two minutes during CPR to prevent fatigue [1]. However, in emergencies, particularly during staff shortages such as pandemics, one rescuer may need to perform extended CPR. This study used a five-minute duration to assess both the two-minute and five-minute intervals and included a 120-minute rest interval based on clinical experience to prevent fatigue accumulation.

The decision to refrain from employing the standing position at the bedside to assess CPR quality was based on well-established evidence indicating that this posture had a significant impact on CPR quality [18]. This effect was especially notable concerning variables such as rescuer height, calf length, bed height, and the use of a taboret during CPR.

### 2.2. Selection of Participants

Participants who met all the following criteria were eligible for inclusion: (1) doctors or nurses in An Nan Hospital; (2) working experience of more than 1 year; and (3) those who had certified advanced cardiovascular life support or basic life support. The exclusion criteria were as follows: (1) those who had a history of spine surgery, sciatica, coronary artery disease, or lung disease such as asthma or chronic obstructive pulmonary disease or were pregnant and (2) those who could not tolerate 2 minutes of CPR. The participants had to sign informed consent forms before joining the study.

### 2.3. Intervention

#### 2.3.1. Choice of N95 Mask

The researchers used the modified ambient aerosol condensation nuclei counter quantitative fit testing protocol (M-QNFT) to test two types of N95 masks before the study: fold-type N95 masks (Champak F550; Taoyuan, Taiwan) and cup-type N95 masks (3 M 1860; St. Paul, MN) (Figures 1(a) and 1(b)). The M-QNFT was performed using the PortaCount Pro+ 8038 Respirator Fit Tester (TSI Inc., Shoreview, MN, USA) according to the OSHA protocol 29CFR 1910.134. Modified ambient aerosol condensation nuclei counter the quantitative fit testing protocol for filtering facepiece respirators [19, 20]. An FF ≥ 200 was scored as 200, and an FF ≥ 100 was considered passing for an N95 respirator. If the N95 mask failed the test in the first round, the researchers taught the participant how to wear it. Ultimately, the researchers chose the mask with the higher pass rate between the two N95 masks as the mask used by all participants.

#### 2.3.2. Type of PPE

The three types of PPE were level D PPE, includes a surgical mask, face shield, hair cover, nitrile gloves, isolation gown, and foot cover (D-PPE); level C PPE, includes an N95 mask, face shield, hair cover, protective clothing (“Ten Quin” Medial Apparel, China), nitrile gloves, foot cover, and isolation gown (C-PPE); and PAPR, including level C PPE plus a PAPR (3 M™ Jupiter™, St. Paul, MN, USA) with a loose-fitting hood (S-433 L-5), breathing tube (BT-20 L), P3 particulate filter, 8-hour battery (5.2 V, NiMH), with an N95 mask inside the hood (Figures 2(a)–2(c)).

#### 2.3.3. Intervention Protocol

With three types of PPE, six different sequences can be drawn for randomization (from A to F) (Figure 3). To ensure that the allocation was concealed, the investigator prepared 6 lots for each sequence, making up a total of 36 opaque sealed lots in one drawing box for the participants to draw the lots. Since all participants had experience donning and doffing C-PPE and PAPR, no further training was performed. At the beginning of the simulation, the investigators provided brief instructions for the overall flow of the study, allowed the participants to complete questionnaires about the demographic characteristics and to provide a baseline subjective visual analog fatigue score, and measured baseline vital signs.

The study was conducted in the pediatric room in the emergency department in this hospital, in which temperature and humidity were controlled at approximately 20∼22°C and 60∼80%, respectively.  Figure 2(d) shows the layout of the test site. The participants knelt on the floor on the left side of the manikin to perform CPR. The PortaCount was placed on the right hand side of the participant, the ambient tube was placed outside the hood, and the inlet of the respirator tube was placed at the N95 mask to continuously monitor the subject's FF. An iPad was placed in front of the participants to show the QCPR SkillReporter app for real-time feedback, and a physiological monitor on the left hand site was used to measure the participants' vital signs before and after CPR.

### 2.4. Outcome Measurements

The primary outcome was the percentage of effective chest compression, which was defined as each chest compression that fit all requirements of the AHA basic life support guidelines [1]. The secondary outcomes were classified into four items. First, FF during the 5 minutes of CPR was continuously monitored. These data were estimated only with C-PPE and PAPR. Second, vital signs, including blood pressure (mmHg), heart rate (beats/min), and pulse oximeter (%) before and after CPR, were recorded by a physiological monitor (Mindray, Taiwan). Third, self-reported subjective visual analog fatigue scores before and after CPR were recorded. A score of 0 means no fatigue at all, while a score of 10 means extreme fatigue [13]. Fourth, the perception of participants while wearing PPE after CPR was assessed. These items were designed and adapted based on considerations from the studies conducted by Park et al. [16] and Ko et al. [17]. This survey had 10 items, including difficulty in donning or doffing the PPE, whether vision was blocked, difficulty breathing, feeling hot while wearing PPE, feelings of fear or anxiety, difficulty communicating, listening, and moving, and difficulty performing CPR. Each item on the survey was scored as 1 = never, 2 = rarely, 3 = sometimes, 4 = most of the time, and 5 = always.

### 2.5. Statistical Method

Based on a pilot study using the “5 min effective chest compressions” factor, the authors estimated that with a significance level of 0.05, a power of 80%, and an effect size of 0.899, a sample size of 12 participants with repeated measurements would be adequate for evaluating the primary outcome. Additionally, we recruited 30 participants with an actual power of 0.91 (91%). Categorical variables are presented as numbers and percentages, and continuous variables are presented as the mean ± standard deviation. Independent *t*-tests were also applied to measure differences between the two groups, and one-way analysis of variance (ANOVA) was used to measure differences between three or more groups, followed by post hoc Bonferroni tests for pairwise comparisons if the ANOVA results were significant. This study applied the McNemar test for repeated measurements between categorical variables. All statistical tests were two-tailed, the level of significance was 0.05, and the analysis was performed using SPSS for Windows, version 17.0 (SPSS Inc., Chicago, USA).

## 3. Results

### 3.1. Basic Characteristics

Thirty-two participants were enrolled in the study, two of whom were excluded due to an inability to complete at least one minute of CPR during the study period. Among the remaining participants, there were 7 physicians and 23 nurses; 16 were male and 14 were female; 80% (24/30) of the participants worked in the emergency department, while the remaining participants worked in the intensive care unit and COVID-19-dedicated ward. The mean, standard deviation, and range of the participants' information were as follows: age, 34.2 ± 5.8 years (25–45 years); working experience, 10.9 ± 5.7 years (2–25 years); height, 168.5 ± 8.5 cm (150–184 cm); weight, 69.7 ± 14.4 kilograms (47–108 kilograms); and body mass index, 24.4 ± 3.8 (17.9–36.5).

### 3.2. Quantitative and Qualitative Tests of the Fit Factor

This study required the M-QNFT to decide which face mask to choose. The M-QNFT scores were significantly higher with the Champak F550 than with the 3 M 1860: bending was 182.6 ± 41.7 vs. 91.8 ± 76.6, *p* < 0.001, talking was 185.8 ± 44.9 vs. 110.2 ± 78.3, *p* < 0.001, head side-to-side was 177.3 ± 47.6 vs. 116.9 ± 72.8, *p* < 0.001 and head up-and-down was 178.2 ± 50.7 vs. 109.3 ± 74.5, *p* < 0.001, respectively. The overall M-QNFT scores were 175.4 ± 51.5 vs. 100.2 ± 75.8, *p* < 0.001. For all participants who wore the face mask in the first round, the pass rate with the Champak F550 was higher than that with the 3 M 1860, 25/30 (83.3%) vs. 14/30 (46.7%), respectively, *p*=0.064 (McNemar test). After the intervention for teaching participants how to wear the mask, the pass rate with the Champak F550 increased to 30/30 (100%), while that with 3M1860 increased only to 18/30 (60%), *p* < 0.001 (McNemar test). Therefore, the researchers chose the Champak F550 as a standard N95 mask in this study.

### 3.3. Effective Chest Compressions with Different Types of PPE

In the analysis of CPR during the first two minutes, the best performance was obtained when using D-PPE, 87.4 ± 0.1%, while C-PPE was 86.2 ± 0.1%, and PAPR was 84.4 ± 0.1%, but there was no significant difference (*p*=0.716). For the entire five-minute evaluation, D-PPE was 82.1 ± 0.2%, C-PPE was 78.4 ± 0.2%, and PAPR was 78.0 ± 0.2%, and these differences in performance still did not reach statistical significance (*p*=0.584) (Figure 4).

### 3.4. FF per Minute between C-PPE and PAPR

C-PPE was worse than PAPR in terms of FF at any particular minute across the five-minute continuous monitoring analysis (Figure 5). The FF of C-PPE vs. PAPR was 188.6 ± 33.6 vs. 200.0 ± 0.0 (*p*=0.011) for the initial two minutes and 183.0 ± 39.9 vs. 198.9 ± 9.2 (*p* < 0.001) for the overall five-minute comparison. However, if an FF ≥ 100 was considered a pass, the C-PPE still met the standard for 96.7% (29/30) in the first two minutes and 86.7% (26/30) in the overall five minutes.

### 3.5. Vital Signs and Fatigue Scores across Different Types of PPE

After 5 minutes of CPR, the participants' systolic blood pressure, diastolic blood pressure, heart rate, and subjective visual analog fatigue score were all increased compared with those before CPR, while the pulse oximeter measured in room air conditions slightly decreased (Table 1). Among these measurements, the heart rate with C-PPE after CPR was significantly higher than that with D-PPE, but the difference in vital signs before and after CPR was not statistically significant. In the fatigue score differences before and after CPR, the values with C-PPE were significantly higher than those obtained in the other two groups.

## 4. Perception of Wearing PPE

Regarding the total scores across the ten items, C-PPE was associated with the worst perception, PAPR was in the middle, and D-PPE was considered the best, and there were significant differences among them (*p* < 0.001). In addition, C-PPE scores were significantly higher than PAPR scores for difficulty breathing, feeling hot while wearing, and difficulty communicating, and PAPR scores were significantly higher than C-PPE scores for donning. For other information, please refer to Table 2.

## 5. Discussion

In studies on the impact of PPE on CPR, the results are conflicting [11–13]. Chen et al. [11] enrolled 40 anesthesia residents in a manikin study without a real-time feedback device and stated that CPR quality deteriorated while wearing level C-PPE. Likewise, Tian et al. [12] enrolled 80 doctors and nurses in another manikin study with a real-time feedback device and concluded that there were significant decreases in chest compression quality in the N95 group versus the surgical mask group. In contrast, Donoghue et al. [13] enrolled 108 participants (nurses, physicians with level C-PPE, and paramedics with level B-PPE) who performed continuous chest compression on a pediatric manikin without a real-time feedback device and showed that the use of PPE did not result in a significant change in CPR quality [13]. In addition, our study concluded that wearing different PPE for five minutes of CPR did not significantly affect the quality of CPR. This was probably because our study used a real-time feedback device during chest compression that has been shown to improve CPR performance during training and in real situations [21], and all participants in our study were physicians and nurses who were experienced in wearing PPE.

Hwang et al. [14] stated that even if the participants passed the QNFT, the N95 respirator did not provide adequate protection against respiratory infections during chest compression. In the Hwang study, 61% of participants who fully passed N95 mask fit testing failed at least one of three sessions of chest compression. In our study, while wearing C-PPE with an N95 mask, only 3.3% (1/30) of the fit tests failed in the first two minutes, and 13.3% (4/30) failed across the entire five-minute evaluation. This was probably due to the use of the fold-type Champak F550, which has a thicker spacer under the metal nose clip to avoid seal leakage, which was quite different from the design compared with cup-type 3 M 1860 (Figures 1(c) and 1(d)). Moreover, past research has shown that FF with fold-type N95 mask is also better than FF with cup-type N95 mask [15].

Regarding the difference in after-CPR and before-CPR, systolic blood pressure, diastolic blood pressure, heart rate, and pulse oximeter remained unchanged among the groups. However, in terms of fatigue scores, the scores with the C-PPE were clearly higher than those with the D-PPE, which was consistent with other studies [11–13]. Interestingly, PAPRs were associated with a significantly lower fatigue score than C-PPE. Therefore, if rescuer fatigue is considered a factor when choosing the type of PPE, PAPRs should be superior to C-PPE.

In a study with 91 participants who wore loose-fitting PAPRs, Park et al. [16] reported that most participants (83%) rarely or never experienced difficulty in verbal communication and only 24% answered that they had difficulty hearing. On the other hand, Ko et al. [17], in a study of prehospital care comparing conventional PPE and PAPRs (with an N95 mask in the hood, similar to our study), found that PAPRs had a negative impact on the overall tasks of CPR (such as chest compression, intubation, and intravenous catheter insertion), while they were more comfortable regarding breathing and thermal stress. However, there seems to be a negative impact on communication and mobility [17]. The abovementioned findings were consistent with our research. Furthermore, participants perceived a negative impact on chest compression quality, but the data revealed no statistically significant difference in CPR quality between the groups this was probably because we tested for chest compression only, but CPR actually includes many actions. In addition, the vision associated with C-PPE was the worst, and it was believed that a face shield outside the N95 mask of C-PPE generates fog and blocks the field of vision during CPR.

Interestingly, at the end of the study, the subjects were asked to wear the C-PPE with the Champak F550 for continuous CPR for one minute and spoke out loudly 1, 2, and 3 to 100 while performing each compression. If FF ≥ 100 was considered a pass, the pass rate of N95 dropped from 100% to 83.3%. Moreover, if FF ≥ 200 was categorized as passing, the pass rate dropped to 43.3% in this minute. Hence, it is not appropriate for rescuers to speak loudly because the face mask will leak around the edges of the respirator, particularly in a rapid ventilation condition.

During the COVID-19 pandemic, infection control supplies have been of paramount importance, yet frequently faced shortages. In an unpublished study conducted by the author's research team in 2023, which investigated the usage of N95 masks among emergency physicians in Taiwan during the pandemic and assessed whether fit testing was performed. The study involved 45 emergency physicians, with 53.3% affiliated with medical centers, 35.6% from regional hospitals, and 11.1% from district hospitals. Notably, the study revealed that 80% of respondents used multiple N95 mask brands, with 17.7% utilizing six or more distinct N95 brands. However, it is concerning that 31.1% of participants disclosed that they had never undergone mask fit testing, while only 15.6% confirmed that all their masks had been subjected to fit testing. These data underscore the frequent brand changes of N95 masks and the inadequate adherence to fit testing protocols, potentially jeopardizing the safety of healthcare workers.

In summary, the results showed that PAPRs were better than C-PPE in terms of the FF, fatigue score, and total perception of wearing, except for doffing. In terms of CPR quality, whether conducted for two minutes or five minutes, there was no significant difference between the PAPRs and C-PPE. Therefore, disregarding cost considerations, the implementation of PAPRs is recommended during CPR to mitigate the risk of aerosol infection. In situations where complete PAPRs' implementation is not feasible, the use of N95 masks with an acceptable FF is a suitable alternative. Additionally, rescuers should refrain from speaking loudly during CPR to minimize the risk of mask leakage, particularly during rapid ventilation.

Nevertheless, our study has several limitations. The manikin is not a real person, and the actions of CPR actually include intubation, electric shock, injection, and drug administration, but we tested only CPR quality. Moreover, certain experts have questioned the necessity of simultaneously using an N95 mask within a PAPR hood. In fact, the N95 mask has proven valuable in situations involving over breathing (inhalation at a flow rate higher than what the PAPR can provide) [22], acting as a contingency plan in the event of PAPR mechanical failure [23], and reducing the risk of contamination during the doffing process of the PAPR. In addition, the utilization of an N95 mask within a PAPR hood does indeed pose limitations, primarily attributed to the height of the N95 mask. This difference is clearly illustrated in Figure 1(b), where the Champak F550 mask measures 9 centimeters in height, while the 3M 1860 mask is only 6 centimeters tall. Remarkably, during the course of this study, one of the participants encountered contact between the mask and the PAPR hood while using the Champak F550 mask. In such circumstances, the use of an N95 mask within the PAPR did not yield benefits.

However, our study also has many advantages; the most important is that it was a very rigorous study design and was quite comprehensive in terms of prognostic parameters. CPR quality, FF, fatigue scores, vital signs, and various aspects of the perception of wearing PPE have not yet been reported in other studies.

## 6. Conclusions

PAPR is recommended when performing CPR in situations where aerosol transmission is suspected. If PAPR cannot be fully implemented, N95 masks with an acceptable FF are recommended for use. Additionally, when using N95 masks, rescuers should avoid speaking loudly during CPR to minimize the risk of mask leakage.

## Figures and Tables

**Figure 1:** The photographs of the 3M 1860 and the Champak F550: (a) frontal view; (b) lateral view; (c) inner view of the 3M 1860; and (d) inner view of the Champak F550.

**Figure 2:** Photos of different types of personal protective equipment (PPE): (a) D-PPE; (b) C-PPE; (c) PAPR; and (d) simulation site of this study.

**Figure 3:** Flowchart for this study.

**Figure 4:** Effective chest compression among different types of PPE.

**Figure 5:** The fit factor per minute between C-PPE and PAPR.

**Table 1:** Comparison of vital signs across different types of personal protective equipment.

	Mean ± standard deviation			*p* value
	D-PPE	C-PPE	PAPR	
Before-systolic blood pressure (mmHg)	121.4 ± 11.5	122.5 ± 13.8	122.7 ± 13.7	0.797
Before-diastolic blood pressure (mmHg)	79.2 ± 8.9	79.9 ± 10.6	80.6 ± 10.2	0.686
Before-heart rate (bpm)	77.2 ± 13.9	80.9 ± 12.2	80.0 ± 11.7	0.102
Before-pulse oximeter (%)	99.3 ± 0.2	99.5 ± 0.2	99.1 ± 0.2	0.072
Before-visual analog fatigue score	2.6 ± 1.6	2.6 ± 1.5	2.5 ± 1.6	0.980
After-systolic blood pressure (mmHg)	135.6 ± 15.9	140.7 ± 17.5	137.7 ± 14.2	0.196
After-diastolic blood pressure (mmHg)	81.0 ± 12.5	82.5 ± 11.2	82.5 ± 12.7	0.609
After-heart rate (bpm)	121.6 ± 17.4	126.9 ± 15.5	123.9 ± 19.1	0.047^*∗*^
After-pulse oximeter (%)	98.9 ± 1.0	98.7 ± 1.1	98.6 ± 1.2	0.626
After-visual analog fatigue score	5.1 ± 1.5	6.4 ± 1.6	5.5 ± 1.3	<0.001^*∗*^^,¶^
Δ-Systolic blood pressure (mmHg)	14.3 ± 12.4	18.1 ± 14.4	14.9 ± 14.1	0.502
Δ-diastolic blood pressure (mmHg)	1.8 ± 8.7	2.6 ± 8.5	1.9 ± 10.2	0.902
Δ-heart rate (bpm)	44.3 ± 15.1	46.0 ± 13.1	43.9 ± 14.8	0.676
Δ-pulse oximeter (%)	−0.4 ± 0.9	−0.7 ± 0.9	−0.3 ± 1.2	0.141
Δ-visual analog fatigue score	2.6 ± 1.3	3.8 ± 1.6	3.0 ± 1.6	<0.001^*∗*^

Δ represents the difference in after-CPR and before-CPR scores. ^*∗*^Significant difference between D-PPE and C-PPE with repeated-measures ANOVA. ^#^Significant difference between D-PPE and PAPR with repeated-measures ANOVA. ^¶^Significant difference between C-PPE and PAPR with repeated-measures ANOVA.

**Table 2:** Perceptions related to wearing different types of personal protective equipment.

	Mean ± standard deviation			*p* value
	D-PPE	C-PPE	PAPR	
Was it difficult to don?	1.5 ± 0.6	2.2 ± 0.7	2.7 ± 0.9	<0.001^*∗*^^,#,¶^
Was it difficult to doff?	1.5 ± 0.5	2.5 ± 0.9	2.8 ± 1.0	<0.001^*∗*^^,#^
Did it obstruct your vision?	2.0 ± 1.0	2.9 ± 0.9	2.8 ± 0.9	0.002^*∗*^^,#^
Was it difficult to breath?	1.9 ± 0.8	3.2 ± 0.8	2.3 ± 0.7	<0.001^*∗*^^,#,¶^
Did it cause you to become hot?	2.6 ± 0.9	3.9 ± 0.9	3.0 ± 1.3	<0.001^*∗*^^,¶^
Did it cause fear and anxiety?	1.5 ± 0.5	2.0 ± 0.8	1.8 ± 0.7	0.008^*∗*^^,#^
Was it difficult to communicate verbally?	1.7 ± 0.6	2.8 ± 0.9	2.3 ± 0.8	<0.001^*∗*^^,#,¶^
Did it lead to difficulty listening?	1.5 ± 0.6	2.3 ± 0.7	2.4 ± 0.8	<0.001^*∗*^^,#^
Did it lead to difficulty moving while performing CPR?	1.9 ± 0.7	3.2 ± 0.8	3.2 ± 0.7	<0.001^*∗*^^,#^
Did it interfere with your ability to do CPR?	1.9 ± 0.7	2.9 ± 0.8	2.7 ± 0.9	<0.001^*∗*^^,#^
Total score of perception	18.0 ± 4.7	27.9 ± 5.4	26.0 ± 5.3	<0.001^*∗*^^,#,¶^

^*∗*^Significant difference between D-PPE and C-PPE with repeated-measures ANOVA. ^#^Significant difference between D-PPE and PAPR with repeated-measures ANOVA. ^¶^Significant difference between C-PPE and PAPR with repeated-measures ANOVA.

## Data Availability

The data used to support the findings of this study are available from the corresponding author upon request.
